The article "Molecular Mechanism of Expression Changes of Immunological Indexes of PD-1/sPD-L1 after Radiotherapy in Nonsmall Cell Lung Cancer" was retracted in 2024. Reasons: signs of a paper mill; compromised peer review; unreliable results or conclusions.

# Molecular Mechanism of Expression Changes of Immunological Indexes of PD-1/sPD-L1 after Radiotherapy in Nonsmall Cell Lung Cancer

**DOI:** 10.1155/2021/8811751

**Published:** 2021-04-20

**Authors:** Yanli Qu, Huan Wang, Hangyu Liu, Xiaohu Sun, Ji Li, Hong Yu

**Affiliations:** Department of Radiation Oncology, Cancer Hospital of China Medical University, Liaoning Cancer Hospital & Institute, Shenyang 110042, China

## Abstract

It is aimed at investigating the changes of serum soluble programmed death-ligand 1 (sPD-L1) expression level in nonsmall cell lung cancer (NSCLC) before and after radiotherapy, the correlation of PD-L1, PD-1, and proteins of Akt (protein kinase B), mTOR, and HIF-1*α*, and the molecular mechanism of the PD-1/PD-L1 pathway in the development of NSCLS. A total of 126 NSCLC patients receiving radiotherapy in Liaoning Cancer Hospital from September 2018 to September 2019 were selected as the observation group, and another 58 healthy volunteers were selected as the control group. NSCLC patients were divided into group A (stage I-II, stereotactic radiotherapy) and group B (stage III, intensity-modulated radiation therapy) according to the cancer stage. The efficacy of radiotherapy was evaluated, and sPD-L1 expression was detected by ELISA. The immunohistochemical staining was adopted to detect protein expressions of Akt, mTOR, and HIF-1*α* in NSCLC tissues. The correlation between their expression and expression of PD-L1 and PD-1 was analyzed. The results showed that the overall response rate (ORR) of group A was 89.29%, the clinical benefit response (CBR) was 96.43%, the median survival time (MST) was 25 months, and the survival rate within three years was 72.56%. In group B, the ORR was 70.41%, the CBR was 97.96%, the MST was 18 months, and the survival rate within three years was 34.67%. Comparison of overall serum sPD-L1 expression in the control group, group A, and group B and between groups before radiotherapy was statistically significant (*P* < 0.01). After radiotherapy, serum sPD-L1 expression in group A and group B decreased compared with that before radiotherapy (*P* < 0.01). Among NSCLC patients, the positive expression rate of Akt, mTOR, and HIF-1*α* was 71.32%, 41.26%, and 80.65%, respectively. PD-L1 expression and Akt, mTOR, and HIF-1*α* expression showed a significant correlation. PD1 expression and Akt, mTOR, and HIF-1*α* expression also showed a significant correlation. It indicated that the expression level of sPD-L1 in NSCLC patients was higher than that in normal subjects, but the expression level of sPD-L1 was decreased after radiotherapy. PD-1/PD-L1 may play important roles in NSCLC procession through the Akt/mTOR and HIF-1*α* pathway.

## 1. Introduction

With the improvement of the economic and the deteriorating living environment, malignant tumors have surpassed cardiovascular diseases as the primary cause of harm to human life and health [1]. Among them, the incidence and mortality of lung cancer rank first among malignant tumors [2]. Lung cancer is mainly divided into two main types: small cell lung cancer and NSCLC. NSCLC accounts for about 80% of all lung cancers [3]. The main clinical treatments for NSCLC include surgery, chemotherapy, radiotherapy, immunotherapy, targeted therapy, and traditional Chinese medicine [4, 5]. Surgery and chemotherapy are usually suitable for the early stages of NSCLC, but usually, 80% of patients are already in the middle and advanced stages when they are diagnosed. And almost half of the patients have distant metastases. The advanced treatment of NSCLC usually adopts chemotherapy or targeted therapy. However, the survival rate of patients in five years after chemotherapy is only 2%, the median survival time is 10 months, and the prognosis effect is poor. Radiotherapy is a local treatment method for tumors, which can be used in different stages and different treatment stages of tumor patients, and the scope of application is very wide [6]. Radiotherapy has become the main clinical treatment for NSCLC.

Studies have shown that tumor cells can escape host immune surveillance by expressing PD-L1 or PD-1 [7]. PD-1 belongs to the CD28 family and consists of 288 amino acids. It plays a key role in tumor immune evasion. PD-L1 is a cooperative signaling molecule that can bind to T cell receptors and can stimulate or inhibit T cell immunity. PD-1/PD-L1 is a very important signal pathway in the tumor microenvironment. It can promote the growth and reproduction of tumor cells and participate in the mediation of immune escape, thereby promoting tumor occurrence and development. Studies showed that after blocking the PD-1/PD-L1 pathway, it shows good antitumor activity during NSCLC treatment [8]. Many studies have revealed that the expression of PD-L1 is closely related to the poor prognosis of lung cancer [9]. The expression level of PD-L1 is an important indicator for evaluating the efficacy of anti-PD-1 or PD-L1 [10]. Studies suggested that Akt-mTOR can regulate the expression of PD-L1 both in vivo and in vitro, and the PD-1/PD-L1 pathway can affect Akt/mTOR oncogene signaling [11]. It indicates that PD-1/PD-L1 may promote tumorigenesis and development through Akt/mTOR pathway. In addition, studies showed that HIF-1*α* may also upregulate PD-L1 expression [12]. Therefore, the changes in serum sPD-L1 levels before and after radiotherapy for nonsmall cell lung cancer were analyzed, so did the correlation of PD-L1 and PD-1 with Akt, mTOR, and HIF-1ɑ proteins, to explore the relevant mechanism of the PD-1/PD-L1 pathway in the occurrence and progression of NSCLS.

## 2. Materials and Methods

### 2.1. Research Subjects and Grouping

A total of 126 NSCLC patients receiving radiotherapy in Liaoning Cancer Hospital from September 2018 to September 2019 were selected as the observation group, and another 58 healthy volunteers were selected as the control group. NSCLC patients were divided into group A (stage I-II, stereotactic radiotherapy) and group B (stage III, intensity-modulated radiation therapy) according to the cancer stage. The trial had been approved by the ethics committee of the Liaoning Cancer Hospital, and all patients included had signed informed consent.

NSCLC inclusion criteria: patients diagnosed with NSCLC; patients with *Eastern Cooperative Oncology Group* (ECOG) performance status score of 0 or 1; IIIA-C patients who had no chemotherapy contraindications and could receive concurrent chemotherapy during radiotherapy; IA3-IIA patients who gave up or refuse surgery.

Inclusion criteria for healthy volunteers: no history of tumor; no infectious disease; no systemic immune disease; no chronic systemic disease; and no trauma or acute infection within 3 months.

### 2.2. Treatment Methods

Patients in group A received stereotactic radiotherapy (Tomo + IMRT). The whole thorax was scanned by four-dimensional positioning CT with a thickness of 1.5 mm. According to CT images and positron emission tomography-computed tomography results, the tumor target area was sketched by physicians, and the planned target volume (PTV) was made. The prescribed dose and dose limits for nearby normal organs were then given. According to the dynamic breathing rhythm, precise stereotactic radiotherapy was started. The prescribed dose of PTV was DT48-60Gy, and the large segmentation irradiation technology was applied, with each dose of 10-15Gy, once a day, and a total of 6 treatments were given. The *α*/*β* ratio was set as 10, and BED was controlled within 90-150Gy.

Patients in group B received intensity-modulated radiation therapy. First, CT positioning was performed. The patient was placed in the supine position, chest enhanced scan positioning was performed, and 3-5 mm layer thickness was set. CT images were obtained from the cricoid cartilage level to the lower boundary of the liver and input into the treatment planning system. Then, the GTV, CTV, and PTVt were outlined. Conventional fractional irradiation was performed using linear accelerator 6MV-X-ray. The dosage requirements were as follows, prescription doses of 60Gy, 2Gy/f/d, 5f/w, and 95% isodose line was used to cover PTV. Finally, concurrent chemotherapy plus sequential chemotherapy was administered. Regimens were etoposide plus cislatin, pemetrexed plus cispatin, and docetaxel plus cisplatin.

### 2.3. Enzyme-Linked Immunosorbent Assay

Fasting blood was collected from all patients, 5 mL peripheral venous blood was collected and centrifuged at 2500 r/min for 10 min after left for 30 min. After centrifugation, the supernatant was kept, labelled, and stored in the refrigerator at -80°C for later use. First, the PD-L1 antibody was diluted to 5 *μ*g/mL. The diluent was 0.05 M pH 9 carbonate coating buffer, 0.1 mL of which was added to each well, and the plate was kept at 4°C overnight. The liquid was removed from the wells, and the plate was washed three times. The sample was diluted 1 : 400 and then added into the reaction wells, left at 37°C for 1 h, and then cleaned. Blank hole, positive control group, and negative control group were set. 0.1 mL enzyme-labelled antibody (dilution after titration) was added to each well, which was placed at 37°C for 30 min to 1 h and cleaned. TMB substrate solution was added and left at 37°C for about 20 min, then, the reaction was terminated. The optical density value was measured at 450 nm with a multifunctional marker. If the optical density value was more than 2.1 times that of the negative control group, it was positive.

### 2.4. Efficacy Assessment

The radiation response was assessed adopting the RTOG acute radiation injury grading standard and the RTOG/EORTC late radiation injury grading standard. The *Response Evaluation Criteria in Solid Tumors* (RECIST) [13] was adopted to evaluate the short-term efficacy. The effects were divided into complete response (CR), partial response (PR), progression of disease (PD), and stabilization of disease (SD). If the lesion disappeared completely and remained for more than one month, it was regarded as CR. If the maximum diameter of tumor decreased by more than 30% and remained for one month, it was regarded as PR. If the tumor increased by more than 20% or new lesions were found, it was regarded as PD. If it is between PR and PD, it was regarded as SD. The short-term response rate (CR + PR) and clinical benefit (CR + PR + SD) were calculated, and MST and survival rate within three years were recorded.

### 2.5. Immunohistochemical Staining

Immunohistochemistry was adopted to detect the Akt, mTOR, and HIF-1*α* in NSCLC tissues. First, tissue sections with a thickness of 4 *μ*m were prepared. They were placed overnight in the oven at 37°C, placed in the oven at 60°C for 2 h, and placed in xylene for 1 h. Then, gradient alcohol hydration treatment was carried out, and the samples were placed in anhydrous ethanol I and anhydrous ethanol II for 15 min, respectively; and in 95%, 85%, and 75% ethanol for 2 min, respectively. Then, the sections were rinsed three times with distilled water. Hydrogen peroxide blocking and antigen retrieval treatment were conducted. Drops of primary and secondary diluent antibodies were added. DAB solution was used for color development, after which the sections were observed under a microscope. Then, the running water was used for the termination of staining. Hematoxylin was added and left for 3 min, and the sections were rinsed with tap water. Differentiated for 2 s in 1% hydrochloric acid alcohol, the sections were rinsed with tap water twice. The final staining results were observed under microscope after adding neutral gum to the slide. The expression results of Akt, mTOR, and HIF-1*α* were evaluated according to the degree of staining and area. Staining area score 0, 1, 2, 3, and 4 corresponded to areas of 0, 0-10%, 10%-50%, 50%-75%, and 75-100%, respectively. Staining degree scores 0, 1, 2, and 3 corresponded to nonstaining, light yellow, brownish yellow, and tan, respectively. The sum of the two was the final score. If the score was above 3 points (including), then, it was positive, while 0-2 was negative.

### 2.6. Statistical Analysis

SPSS 20.0 software was adopted for statistical analysis. The measurement data were expressed as mean plus or minus standard deviation ($\bar{x}\pm s$), and *t*-test was adopted for comparison between groups. The counting data were expressed as percentage (%), and chi-square test was used for comparison between groups. Correlation analysis was conducted via rank sum test. *P* < 0.05 was considered statistically significant.

## 3. Results

### 3.1. Comparison of Basic Data of Patients

A total of 184 subjects were selected, including 126 NSCLC patients receiving radiotherapy (observation group) and 58 healthy physical examination personnel (control group). The basic data were shown in Table 1. There were 58 volunteers in the control group, including 38 males and 20 females, with an average age of 62.76 ± 12.53 years old. There were 17, 2, 10, and 29 patients who had never smoked, occasionally smoked, smoked no more than 500 cigarettes per year, and smoked more than 500 cigarettes per year. The patients with ECOG score of 0, 1, and 2 were 58, 0, and 0, respectively. There were 126 patients in the observation group, including 89 males and 37 females, with an average age of 65.39 ± 10.12 years old. There were 25, 11, 35, and 55 patients who never smoked, occasionally smoked, smoked no more than 500 cigarettes per year, and smoked more than 500 cigarettes per year. The patients with ECOG score of 0, 1, and 2 were 2, 43, and 81, respectively.

Patients in the observation group were divided into two subgroups A and B according to different tumor stages, and the basic data of patients in the two groups were shown in Table 2. There were 28 patients in group A, including 19 males and 9 females, with an average age of 71.65 ± 11.36 years old. There were 4, 2, 8, and 14 patients who never smoked, occasionally smoked, smoked no more than 500 cigarettes per year, and smoked more than 500 cigarettes per year. Patients with ECOG score of 0, 1, and 2 were 2, 19, and 7, respectively. There were 16 cases with squamous cell carcinoma and 12 cases with adenocarcinoma. There were 98 patients in group B, including 66 males and 32 females, with an average age of 60.38 ± 10.34 years old. There were 21, 9, 27, and 41 patients who had never smoked, occasionally smoked, smoked no more than 500 cigarettes per year, and smoked more than 500 cigarettes per year. Patients with ECOG score of 0, 1, and 2 were 0, 24, and 74, respectively. There were 48 cases with squamous cell carcinoma and 40 cases with adenocarcinoma.

### 3.2. Evaluation of Therapeutic Effects

The efficacy evaluation results of the two groups were shown in Figure 1. In group A, there were 5 patients with CR, 20 patients with PR, 2 patients with SD, and 1 patient with PD. The ORR was 89.29%, the CBR was 96.43%, the MST was 25 months, and the survival rate within three years was 72.56%. In group B, there were 0 patients with CR, 69 patients with PR, 27 patients with SD, and 2 patients with PD. The ORR was 70.41%, the CBR was 97.96%, the MST was 18 months, and the survival rate within three years was 34.67%. In comparison, group A had an advantage over group B, which was related to the tumor stage. The baseline imbalance between the two groups made it impossible to compare the differences in the efficacy of the two radiotherapy techniques at this level.

### 3.3. sPD-L1 Level before Radiotherapy

The serum sPD-L1 expression levels of all subjects before radiotherapy were shown in Table 3. The serum sPD-L1 expression level of the control group was 176.56 pg/mL (163.23, 183.56), and that in group A and B was 185.76 pg/ml (179.87, 190.35) and 206.18 pg/mL (194.63, 218.68), respectively. Kruskal-Wallis *H* and Mann–Whitney *U* were adopted to conduct significance test. The expression levels of serum sPD-L1 among the three groups and between the two groups were statistically significant (*P* < 0.01). The receiver operating characteristic (ROC) curve of serum sPD-L1 expression of all subjects before radiotherapy was shown in Figure 2. The area under the curve was 0.85, the specificity was 0.765, and the sensitivity was 0.772. Therefore, serum sPD-L1 expression could be taken as a diagnostic indicator for NSCLC.

### 3.4. Changes in sPD-L1 Levels after Treatment

The serum sPD-L1 expression levels of patients in group A and group B after radiotherapy were shown in Tables 4 and 5, respectively. Serum sPD-L1 expression levels were significantly lower in group A 2 weeks and 3 months after radiotherapy than before. Furthermore, rank-sum test showed that there were significant differences in serum sPD-L1 expression level in group A before and after radiotherapy (*P* < 0.01). The expression level of serum sPD-L1 in group B was significantly decreased after radiotherapy, which was the lowest at the 6th week and increased at the 3rd month. However, compared with group A before radiotherapy, the expression level of serum sPD-L1 decreased. Moreover, rank-sum test showed that there were significant differences in serum sPD-L1 expression level in group B before and after radiotherapy (*P* < 0.01).

### 3.5. Expressions of PD-1 and PD-L1

The expression of PD-1 and PD-L1 in tumor cells, cancer mesenchymal cells, and tumor-infiltrating lymphocytes was shown in Figure 3. PD-L1 was found in tumor cells and cancer mesenchymal cells, while PD-1 was expressed in tumor-infiltrating lymphocytes. In all NSCLC patients, the positive expression rate of PD-L1 in lung cancer cells and cancer mesenchymal cells was 59.56% and 64.35%, and the positive expression rate of PD-1 in tumor-infiltrating lymphocytes was 43.67%.

### 3.6. Expressions of Akt, mTOR, and HIF-1*α*

The expression of Akt, mTOR, and HIF-1*α* in NSCLC tissue was shown in Figure 4. Akt was expressed in the nucleus and cytoplasm, mTOR was expressed in the cytoplasm, and HIF-1*α* was expressed in the nucleus. The positive expression of Akt, mTOR, and HIF-1*α* in NSCLC patients was shown in Figure 5. In all NSCLC patients, the positive expression rate of Akt was 71.32%, the positive expression rate of mTOR was 41.26%, and the positive expression rate of HIF-1*α* was 80.65%.

### 3.7. Correlation of PD-1 and PD-L1 with Akt, mTOR, and HIF-1*α*

The collection of PD-L1 with Akt, mTOR, and HIF-1*α* was shown in Figure 6. The expression rates of PD-L1 in Akt-positive and negative patients were 65.45% and 41.87%, respectively. The expression rate of PD-L1 in Akt-positive patients was significantly higher than that of Akt-negative patients, *P* < 0.05. The expression rates of PD-L1 in patients with positive and negative mTOR expression were 71.32% and 51.45%, respectively. The PD-L1 expression rate in mTOR-positive patients was significantly higher than that in mTOR-negative patients, *P* < 0.05. The expression rates of PD-L1 in HIF-1*α* positive and negative patients were 63.83% and 31.56%, respectively. The PD-L1 expression rate in HIF-1*α*-positive patients was significantly higher than that in HIF-1*α*-negative patients, *P* < 0.05.

The collection of PD-1 with Akt, mTOR, and HIF-1*α* was shown in Figure 7. The expression rate of PD1 in Akt positive and negative patients was 51.26% and 27.54%, respectively. The PD1 expression rate in Akt-positive patients was significantly higher than that in Akt-negative patients, *P* < 0.05. The expression rates of PD1 in mTOR positive and negative patients were 54.65% and 33.18%, respectively. The PD-L1 expression rate in mTOR positive patients was significantly higher than that in mTOR negative patients, *P* < 0.05. The expression rate of PD1 in HIF-1*α* positive and negative patients was 48.76% and 21.61%, respectively. The PD1 expression rate in HIF-1*α* positive patients was significantly higher than that in HIF-1*α* negative patients, *P* < 0.05.

## 4. Discussion

Lung cancer is a common malignant tumor, and it is difficult to cure because it is usually found in the advanced stage. The clinical efficacy of radiotherapy in NSCLC patients was evaluated. It was found that the ORR of the stereotactic radiotherapy group was 89.29%, the CBR was 96.43%, the MST was 25 months, and the survival rate within three years was 72.56%. In the intensity-modulated radiation therapy group, the ORR was 70.41%, the CBR was 97.96%, the MST was 18 months, and the survival rate within three years was 34.67%. This was almost consistent with the results of studies of Videtic et al. (2017) [14]. ELISA was adopted to detect the changes in the serum sPD-L1 level of patients, and it was found that the sPD-L1 expression level of NSCLC patients was higher than that of normal people, which showed a downward trend after radiotherapy. It was suggested that the level of sPD-L1 could predict the efficacy of radiotherapy in patients. In the treatment of NSCLC, the change of sPD-L1 as a predictive indicator had great clinical guiding significance [15].

Malignant tumor cells can upregulate immunosuppressive factors or immune checkpoints, thereby exempting themselves from the surveillance of the host's immune surveillance system and thus will not be eliminated by the body [16]. If the expression of tumor cell PD-L1/2 and T cell PD-1 is increased, the T cell-mediated immune surveillance system can be suppressed, and tumor cells continue to survive. If the signal is suppressed, the body's immune system is activated, and then tumor cells are eliminated. This study showed that in NSCLC patients, the positive expression rate of Akt was 71.32%, the positive expression rate of mTOR was 41.26%, and the positive expression rate of HIF-1*α* was 80.65%. This was consistent with the results of Guo et al. (2019) [17]. The expression of PD-L1 and PD1 was both significantly correlated with the expression of Akt, mTOR, and HIF-1*α*, indicating that PD-1/PD-L1 may play an important role in the pathogenesis of NSCLC through Akt/mTOR and HIF-1*α* pathways, but the related mechanisms still needed to be further studied.

## 5. Conclusion

Serum sPD-L1 expression level of NSCLC patients before and after radiotherapy was detected. It was found that the expression level of sPD-L1 in NSCLC patients was higher than that in normal subjects, and the level of sPD-L1 showed a downward trend after radiotherapy. Then, an analysis of the correlation of PD-L1 and PD-1 with Akt, mTOR, and HIF-1*α* was conducted. Results showed that the PD-1/PD-L1 may play important roles in NSCLC procession through the Akt/mTOR and HIF-1*α* pathway. However, there are still some deficiencies in this study, including the limited number of subjects and limitations of immunohistochemistry detection technology. Therefore, the number of samples will be increased in the future, and prospective randomized controlled trials will be conducted to further explore the related mechanism of PD-L1 or PD1 expression in NSCLC. In summary, the study results provided new ideas for the clinical treatment of NSCLC.

## Figures and Tables

**Figure 1:** Comparison of radiotherapy efficacy between the two groups. ((a) was the evaluation result of RECIST; (b) was ORR and CBR; (c) was the MST; (d) was survival rate within three years).

**Figure 2:** ROC curve of serum sPD-L1 expression before radiotherapy of all subjects.

**Figure 3:** The immunohistochemical results of PD-1 and PD-L1 (SP × 200). (a–c) were tumor cells, cancer mesenchymal cells, and tumor-infiltrating lymphocytes, respectively. A1 was PD-L1 (negative); A2 was PD-L1 (positive); B1 was PD-L1 (negative); B2 was PD-L1 (positive); C1 was PD-1 (negative); C2 was PD-1 (positive).

**Figure 4:** Immunohistochemical results of Akt, mTOR, and HIF-1*α* in NSCLC tissues (SP × 200). (A1 was Akt (negative); A2 was Akt (positive); B1 was mTOR (negative); B2 was mTOR (positive); C1 wasHIF-1*α* (negative); C2 wasHIF-1*α* (positive)).

**Figure 5:** The expression of Akt, mTOR, and HIF-1*α* in NSCLC patients.

**Figure 6:** Correlation of PD-L1 with Akt, mTOR, and HIF-1*α*. ((a) was Akt; (b) was mTOR; (c) was HIF-1*α*).

**Figure 7:** Correlation of PD-1 with Akt, mTOR, and HIF-1*α*. ((a) was Akt; (b) was mTOR; (c) was HIF-1*α*).

**Table 1:** Basic data of patients in the control group and observation group.

		Control group (*n* = 58)	Observation group (*n* = 126)	*P*
Gender (male/female)		38/20	89/37	>0.05
Age (years)		62.76 ± 12.53	65.39 ± 10.12	<0.05
Smoking status (person)	Never	17	25	>0.05
	Occasionally	2	11	
	No more than 500 cigarettes per year	10	35	
	More than 500 cigarettes per year	29	55	
ECOG scores	0	58	2	<0.01
	1	0	43	
	2	0	81	

**Table 2:** Basic data of NSCLC patients.

		Group A (*n* = 28)	Group B (*n* = 98)	*P*
Gender (male/female)		19/9	66/32	>0.05
Age (years)		71.65 ± 11.36	60.38 ± 10.34	<0.05
Smoking status (person)	Never	4	21	>0.05
	Occasionally	2	9	
	No more than 500 cigarettes per year	8	27	
	More than 500 cigarettes per year	14	41	
ECOG scores	0	2	0	>0.05
	1	19	24	
	2	7	74	
Pathological type (number of persons)	Adenocarcinoma	12	50	>0.05
	Squamous cell carcinomas	16	48	

**Table 3:** Serum sPD-L1 expression levels of all subjects before radiotherapy (median (25% quantile, 75% quantile)).

	Control group	Group A	Group B
sPD-L1expression level	176.56 pg/mL (163.23, 183.56)	185.76 pg/mL (179.87, 190.35)	206.18 pg/mL (194.63, 218.68)

**Table 4:** Serum sPD-L1 expression level in group A after radiotherapy (median (25% quantile, 75% quantile)).

	0 day	2 weeks	3 months
Group A	185.76 pg/mL (179.87, 190.35)	176.52 pg/mL (166.54, 178.32)	165.78 pg/mL (160.87, 176.23)

**Table 5:** Serum sPD-L1 expression level in group B after radiotherapy (median (25% quantile, 75% quantile)).

	0 day	2 weeks	4 weeks	6 weeks	3 months
Group B	206.18 pg/mL (194.63, 218.68)	200.98 pg/mL (189.56, 213.67)	182.56 pg/mL (172.78, 191.81)	165.56 pg/mL (161.98, 174.93)	185.23 pg/mL (170.29, 200.64)

## Data Availability

All data, models, and code generated or used during the study appear in the submitted article.
